# Computational Methods for Physiological Signal Processing and Data Analysis

**DOI:** 10.1155/2022/9861801

**Published:** 2022-08-10

**Authors:** Yunfeng Wu, Sridhar Krishnan, Behnaz Ghoraani

**Affiliations:** ^1^School of Informatics, Xiamen University, 422 Si Ming South Road, Xiamen, Fujian 361005, China; ^2^Department of Electrical, Computer, And Biomedical Engineering, Toronto Metropolitan University, 350 Victoria Street, M5B2K3, Toronto, ON, Canada; ^3^Department of Computer and Electrical Engineering and Computer Science, Florida Atlantic University, Boca Raton, FL 33431, USA

## Abstract

Biomedical signal processing and data analysis play pivotal roles in the advanced medical expert system solutions. Signal processing tools are able to diminish the potential artifact effects and improve the anticipative signal quality. Data analysis techniques can assist in reducing redundant data dimensions and extracting dominant features associated with pathological status. Recent computational methods have greatly improved the effectiveness of signal processing and data analysis, to support the efficient point-of-care diagnosis and accurate medical decision-making. This editorial article highlights the research works published in the special issue of Computational Methods for Physiological Signal Processing and Data Analysis. The context introduces three deep learning applications in epileptic seizure detection, human exercise intensity analysis, and lung nodule CT image segmentation, respectively. The article also summarizes the research works on detection of event-related potential in the single-trial electroencephalogram (EEG) signals during the auditory tests, along with the methodology on estimating the generalized exponential distribution parameters using the simulated and real data produced under the Type I generalized progressive hybrid censoring schemes. The article concludes with perspectives and discussions on future trends in biomedical signal processing and data analysis technologies.

## 1. Introduction

Nowadays, most point-of-care healthcare systems consist of several biomedical sensors to acquire physiological signals and data to support health condition monitoring and early-stage pathology screening functions [1]. Integration and fusion of the massive multiscale biomedical signals recorded by wearable sensors or medical images generated by multiple imaging modalities have attracted more and more attentions from the research community [2–4]. Advanced computational tools can be effectively used to compute signal dynamics, time-frequency properties, data correlations, and statistical parameters for understanding the complex physiological processes associated with disease symptoms. The emerging deep learning neural networks and machine learning algorithms have the advantages of representing high-dimensional data features with hierarchical network layers, and achieving the accurate pattern classification results, which helps provide the informative diagnostic references for medical decision-making in clinical applications. This special issue collects several research works on the topic of computational methods for physiological signal processing and data analysis, which are summarized as follows.

### 1.1. Time-Frequency Analysis and Deep Learning for Epileptic Seizure Detection

Epilepsy is a type of neurological disorder characterized by the recurring seizures due to sudden surges of disturbed electrical activities in the brain [5]. Patients with epilepsy commonly suffer from involuntary convulsions, a loss of consciousness, and other movement disorders [6]. The electroencephalogram (EEG) records the potentials of cerebral cortex based on the electrodes attached to the scalp, which may manifest the electrical activities in the brain. Detection of epileptic seizure using only a single-channel EEG signal is a challenge, because such a task should explore the limited information from the single-channel signal, and construct an effective system with acceptable classification accuracy and robustness as well.

In [7], Pan et al. first studied the temporal waveform variants of the single-channel EEG signals of patients with epilepsy, along with the frequency-domain properties based on the discrete Fourier transform (DFT). Then, they implemented the signal segmentations with multiple fixed-length windows and characterized the time-varying changes of frequency components in the EEG signals using the discrete wavelet transform and short-time Fourier transform [7]. The time-domain, frequency-domain, and time-frequency features were fused as a hybrid representation of the epileptic EEG signals. Four well-devised convolutional neural networks (CNNs) were employed to accomplish the signal classification task. Pan et al. [7] considered the “divide-and-conquer” strategy and sent each EEG feature to an individual lightweight CNN. Each CNN was regularized with reduced parameters to perform the depthwise convolution and pointwise convolution operations and output the patterns through the maximum pooling layer. The syncretic patterns were finally combined to detect the epileptic seizure events. The results evaluated with 5-fold, 10-fold, and 20-fold cross-validation methods demonstrated that the hybrid time-frequency features and deep learning neural networks can improve the accuracy performance in the epileptic seizure detection [7].

### 1.2. ERP Latency Detection in Single-Trial EEG Signals

Detection of amplitude and latency components in a single-trial EEG signal requires a series of artifact removal, feature extraction, and event-related potential (ERP) identification procedures. In [8], Zang et al. developed an effective machine learning technique for latency detection in single-trial EEG signals, instead of the conventional superposition and average method. Two different EEG data sets (i.e., simulated N170 and real P50 recordings) were tested for the performance evaluation purpose. The simulated EEG signals with N170 ERP components were obtained from the benchmark data set of Texas State University, USA. A total of 21 young subjects repeated 4 min eyes closed and 4 min eyes open behaviors in a resting state. The 72-channel EEG signals were downsampled to 256 Hz for subsequent pattern analysis. The real single-trial ERP data were recorded from 8 subjects who performed the 15 min auditory tests with three delayed-response tasks.

In order to improve the EEG signal quality, Zang et al. [8] implemented the signal preprocessing procedures to remove artifacts. The low-frequency noise was first eliminated using a high-pass finite impulse response (FIR) filter (with the cutoff frequency at 1 Hz). The electroocular artifacts, blinks, and baseline shifts were cancelled using the EEGLAB toolbox. Then, the single-trial EEG signals were segmented into several fixed-length epochs, with the linked mastoids as references.

The logistic regression, multilayer perceptrons, and support vector machine classifiers were utilized to distinguish the ERP latency components in each epoch. The experimental results showed that the multilayer perceptrons was able to provide an accuracy up to 90.69% of N170 latencies on the simulated data set. The method proposed by Zang et al. [8] significantly outperformed the Woody filter in different signal-to-noise (SNR) conditions. The experimental results on the real ERP data set indicated that the P50 amplitudes evoked by the first sound were significantly larger than those evoked by the second sound in three auditory tasks. Such results were consistently reproduced until the ending of sensory gating, which showed an excellent generalization capability.

### 1.3. Analysis of Athlete Exercise Intensity with ECG and PCG

The physiological signals are useful for monitoring and assessing the physical status of athletes. Wang and Zhu carried out an interesting research work on monitoring and categorizing the body exercise intensity conditions by means of electrocardiogram (ECG) and phonocardiogram (PCG) signal analysis [9]. The ECG and PCG signals were first projected onto an image with various motion intensity annotations. The AlexNet CNN architecture that contained five conventional layers, one pooling layer, and three fully connected layers was employed to perform the classifications of body exercise intensities of athletes [9]. With the purpose of visualizing the cluster scatters, the t-SNE technique was used to reduce the data dimensions in the fully connected layers of the AlexNet architecture. The exercise intensity patterns include the human activities during bicycle, treadmill, stationary bicycle, walking at constant speed, laying on bed, and sitting on armchair [9]. The classification results indicated that the AlexNet was able to provide the highest overall accuracy (95.7%) for six types of exercise intensity [9], which was superior to the results reported in the previous related works.

### 1.4. Lung Nodule CT Image Segmentation and Detection Based on Multiposition U-Net

Caused by different respiratory disorders and infections, lung (pulmonary) nodules would grow in the form of small abnormal masses in the lung. Lung nodules can be detected and diagnosed as begin or cancerous using the computed tomography (CT) imaging technique. Automatic segmentation and detection of the lung nodule regions from the CT scanned images could greatly reduce the radiologists' workload and also provide informative references for further accurate diagnosis in clinical practice.

The major contributions of Zhang et al. [10] focused on three parts, i.e., lung parenchyma segmentation, extraction of lung nodule regions, and sign classification based on CT image morphological features. The U-shape network (U-Net) paradigm was utilized to accomplish these three tasks. In the lung parenchyma segmentation procedure, the attention mechanism was applied to prevent the background pixel interferences and ameliorate the semantic segmentation accuracy of the U-Net [10]. Then, the regions of interest can be localized from the receptive fields with the dense atrous convolution approach. A dense connected block module was used to reduce the network parameters and avoid the redundant convolution computations. In the lung nodule extraction and sign classification procedures, the Mish activation function was used to speed up the network transmission durations and improve the computation efficiency. A two-way enhanced feature pyramid network was employed to integrate the low-level pixel features and high-level semantic features through the two-way cross-scale connections. The classification results indicated that the unified U-Net method proposed by Zhang et al. [10] may achieve the best sensitivity (91%) and specificity (88%) values and the excellent receiver operating characteristic curve, in comparison with the other traditional machine learning algorithms.

### 1.5. Estimation of Maximum Likelihood and Bayesian Model Parameters

Statistical models are useful to describe the nonstationary random process of electrophysiological signals. The parameters of probability distribution estimators should be properly calculated from the data observations in long-term experiments. The Type I generalized progressive hybrid censoring scheme comprehensively considers both of the Type I and Type II data censoring scenarios.

In [11], Nagy and Alrasheedi presented the methods for estimating the parameters of maximum likelihood and Bayesian estimators, based on the Type I generalized progressive hybrid censored data. They first described the probability density and cumulative distribution functions of a generalized exponential distribution. Then, the Type I progressive censoring data generated from the generalized exponential distribution were used to compute the shape and scale parameters for estimating the maximum likelihood models. The following text presented the statistical inference procedures for approximating the confidence intervals for the shape and scale parameters, respectively. Confidence intervals for the reliability function and hazard functions of the maximum likelihood estimators were calculated using the delta method.

Nagy and Alrasheedi [11] also discussed the Bayesian estimates of the shape and scale parameters of the generalized exponential distribution. The generalized progressive hybrid censoring scheme data were generated with the Markov chain Monte Carlo approach and the Gibbs sampling procedure. In addition, Nagy and Alrasheedi [11] computed the reliability and hazard functions and their credible intervals for the generalized exponential distribution based on the real deep groove ball bearings data. They concluded that the Bayesian estimates of the shape and scale parameters would bring smaller mean squared errors with the combination of Type I and Type II progressive hybrid censored data [11].

### 1.6. Memory Activity Classification Based on EEG Signal Analysis

The changes of memory activities in the brain can be measured and recorded by EEG signals. In [12], Xi et al. studied the classifications of memory activities with different memory loads or targets based on EEG signal analysis. The memory task experiments simultaneously acquired the 32-lead EEG signals and the corresponding behavioral data from 19 healthy subjects. The preprocessing and reduction of mode interferences were implemented using the independent component analysis (ICA) method.

A 4th-order Butterworth filter was used to extract the EEG components of Gamma rhythm at 30–100 Hz [12]. Then, the extract signal components of Gamma rhythm were segmented with 1 s durations immediately prior to each valid finger clicking moment. The phase locking value of Gamma rhythm between each pair of leads was estimated, and the binarization was determined based on a threshold of 0.179 based on a band-pass filter [12]. The brain network characteristics were computed with the binarized phase locking values, and a support vector machine with radial basis function kernels was used to classify the memory activities. The experimental results showed that the brain network characteristics of node degree, local clustering coefficient, and betweenness centrality were useful for classifications of the presence or absence of memory and analysis of the mental workload intensity at the moment of memory [12].

## 2. Perspectives

With the development of wearable biosensors, the volume and dimensions of biomedical signals and images have extensively increased. Raw data records are very susceptible to random noise and external interferences. Novel signal processing and analysis techniques can eliminate the artifacts and guarantee the signal quality for pattern analysis.

The state-of-the-art signal feature analysis literature mainly focuses on time-domain, frequency-domain, joint time-frequency domain, and sparse signal feature extractions [13]. The temporal waveform changes can be parameterized with linear regression and autoregressive models.

The frequency features can be computed with the power spectral density derived from the discrete cosine transform and fast Fourier transform. The frequency variants with respect to different time spans can be characterized by the continuous wavelet transform, short-time Fourier transform, and wavelet packet transform [13]. The research work of Zang et al. [8] has demonstrated the merits of joint time-frequency features in the epileptic seizure detection application.

Recently, the international research community has emphasized the sparse signal decomposition and reconstruction. The representative works are the empirical mode decomposition [14] and singular value decomposition [15]. The artifacts and signal components can be separated into different channels during the iterative computation processes [16]. The sparse signal representations can be used as the distinct features for further pattern classifications.

Deep learning neural networks are prevailing in medical diagnosis applications nowadays [17]. The deep learning networks are commonly composed of several convolution, pooling, and fully connected layers, which can better cope with the spatial features in high-dimensional spaces. The reduction of unnecessary network parameters and construction of hybrid network combinations are the future trends in deep learning.
